# Revealing an association between HPV and systemic lupus erythematosus: A bidirectional two‐sample Mendelian randomization study

**DOI:** 10.1111/srt.13913

**Published:** 2024-08-07

**Authors:** Fangfang Pan, Huiliang Shen, Ben Wang, Jian Wang

**Affiliations:** ^1^ Department of Gynecology Zhejiang Dermatology Hospital Huzhou Zhejiang China; ^2^ Department of Dermatology Zhejiang Dermatology Hospital Huzhou Zhejiang China; ^3^ Department of Information Technology Zhejiang Dermatology Hospital Huzhou Zhejiang China

**Keywords:** Genome‐wide association studies, HPV 16/18, Human papillomavirus, Systemic lupus erythematosus, Two‐sample Mendelian Randomization study

## Abstract

**Background:**

An increasing number of studies have focused on the association between Human papillomavirus (HPV) infection and systemic lupus erythematosus (SLE). However, current evidence is largely based on retrospective studies, which are susceptible to confounding factors and cannot establish causation.

**Methods:**

A bidirectional two‐sample Mendelian randomization (MR) design was used to evaluate the causal relationship between HPV and SLE. Mononucleoside polymers (SNPS) with strong evidence for genome‐wide association studies (GWAS) were selected from the HPV exposure dataset and used as an instrumental variable (IV) for this study. For the MR Analysis results, the MR‐Egger intercept P test, MR‐Presso global test, CochranQ test and leave‐one test were used for sensitivity analysis.

**Results:**

Based on the evidence of MR Analysis, this study finally determined that there was no causal association between HPV16 and HPV18 and SLE.

**Conclusions:**

Possible regulation of HPV infection is not significantly associated with regulation of SLE. These findings provide new insights into the underlying mechanisms of HPV and SLE and need to be validated by further studies.

## 1 INTRODUCTION

Systemic lupus erythematosus (SLE) is a chronic autoimmune disease marked by widespread inflammation and tissue damage.^1^ Its etiology is complex, involving genetic, environmental, and hormonal factors. Among the environmental contributors, infectious agents like viruses have been implicated in the development of autoimmune diseases.^2^, ^3^ Human papillomavirus (HPV), primarily known for causing cervical and other cancers, has also been suggested as a potential contributor to autoimmune conditions, including SLE.^4^, ^5^

While numerous studies have explored the association between HPV infection and SLE, most have been retrospective, thus limiting their ability to establish causation due to potential confounding factors.^6^, ^7^, ^8^ To overcome these limitations, a more rigorous methodological approach is necessary to investigate the potential causal link between HPV and SLE.

Mendelian randomization (MR) is an epidemiological technique that employs genetic variants as instrumental variables (IVs) to assess the causal effect of an exposure on an outcome.^9^ This method helps to address confounding and reverse causation issues inherent in observational studies. In this study, we utilized a bidirectional two‐sample MR design to evaluate the causal relationship between HPV and SLE, drawing on genome‐wide association study (GWAS) data for both HPV exposure and SLE outcomes.

By leveraging genetic variants as proxies for HPV infection and performing MR analysis, we aimed to provide clearer insights into whether HPV contributes to the development of SLE or vice versa. Our findings have the potential to significantly enhance our understanding of the mechanisms linking viral infections and autoimmune diseases, and to inform the development of preventive and therapeutic strategies.

## 2 METHOD

### 2.1 GWAS summary data of exposure and outcome

The HPV 16/18 protein exposure dataset was downloaded from the MRC IEU OpenGWAS (https://gwas.mrcieu.ac.uk/), a European population assay of 1124 plasma proteins quantified in the GWAS study. The HPV16/18 E7 protein was included in the assay of 1124 plasma proteins. SLE data were obtained from a European population cohort consisting of 647 SLE patients and 482 264 controls.

### 2.2 Statistical analysis

Genetic variants were selected as IVs if reaching the genome‐wide significance (GWAS *p*‐value < 5e − 05) and were further clumped based on linkage disequilibrium (LD, *r* ^2^ = 0.001) and genomic region (clump window 10 000 kilobases). The inverse variance weighted (IVW), MR‐Egger, weighted median, simple mode and weighted mode are the major MR analysis methods to confirm robust results, and IVW was used as the major analysis as random‐effect model.

Sensitivity analyses were pivotal in MR studies to provide robust causal inferences under weaker assumptions. We applied Cochran *Q* test to assess heterogeneity. Meanwhile, test for interception in MR‐Egger can identify and control bias due to horizontal pleiotropy. Specifically, Steiger directional tests were adopted to assess reverse causality.

All analyses were performed using the R statistical software version 4.3.1 with the two sample MR and forest plotter (https://github.com/adayim/forestploter) packages.

## 3 RESULTS

### 3.1 HPV 16/18 genetic variable screening

We identified 23 SNPS in HPV16 by association analysis (*p* < 5e − 05) and linkage disequilibrium analysis (kb = 10 000, *r* ^2^ = 0.001) followed by the removal of weak instrumental variables (Figure 1A, *F* > 10). Thirteen SNPS were identified in HPV18 type (Table S1), which were used as valid IVS for subsequent MR Analysis (Figure 1B).

**FIGURE 1:** HPV‐associated SNP screening. (A) HPV16‐related SNPS. (B) HPV18‐related SNPS.

### 3.2 MR analysis of HPV 16/18 and SLE

We conducted MR analysis of the SNP selected above and SLE to identify the causal association between HPV and SLE. Our results showed that there was no causal association between HPV16 and SLE (OR = 0.964, 95%CI: 0.866–1.074; *p* = 0.506, Figure 2A), in addition, there was no causal association between HPV18 and SLE (OR = 0.958, 95% CI: (0.840–1.092; *p* = 0.521, Figure 2B). In order to verify the reliability of the results, we conducted heterogeneity and sensitivity tests, and found that the Q values of HPV16/18 were 0.124 and 0.693, respectively. In addition, the values of sensitivity check were 0.678 and 0.279, indicating that the results were reliable.

**FIGURE 2:** MR analysis results. (A) MR analysis of HPV16 and SLE. (B) MR analysis of HPV18 and SLE. (C) Reverse MR analysis of HPV16 and SLE. (D) Reverse MR analysis of HPV18 and SLE.

### 3.3 Reverse MR analysis of HPV 16/18 and SLE

We conducted a bidirectional Mendelian randomization study to further explore the causal association between SLE and HPV16/18, and our results showed no causal association between SLE and HPV16 (OR = 1.058, 95% CI: 0.967 – 1.157; *p* = 0.218, Figure 2C), and there was no causal association between SLE and HPV18 (OR = 1.015, 95% CI: (0.893 – 1.153; *p* = 0.820, Figure 2D). In order to verify the reliability of the results, we conducted heterogeneity and sensitivity tests, and found that the *Q* values of HPV16/18 were 0.480 and 0.006, respectively. In addition, the sensitivity test values were 0.184 and 0.999, indicating bias in SLE and HPV18. However, the results proved to be reliable in sensitivity analysis.

## 4 DISCUSSIONS

In this study, we employed a bidirectional two‐sample Mendelian randomization (MR) approach to investigate the potential causal relationship between human papillomavirus (HPV) infection and systemic lupus erythematosus (SLE). Our analysis found no evidence of a causal association between HPV16 or HPV18 and SLE, nor between SLE and these HPV types.

Our findings suggest that HPV infection does not causally influence the development of SLE, nor does SLE predispose individuals to HPV infection. These results are consistent with some previous observational studies that have failed to establish a clear link between viral infections and autoimmune diseases. However, our study benefits from the MR approach, which helps to mitigate confounding factors and reverse causation that often plague observational studies.

One of the strengths of our study is the rigorous methodological approach.^10^, ^11^ The bidirectional MR design allows us to test for causality in both directions, providing a comprehensive assessment of the relationship between HPV and SLE. Additionally, the use of large‐scale GWAS datasets for both HPV exposure and SLE outcomes enhances the robustness and reliability of our findings. Multiple sensitivity analyses, including the Cochran Q test for heterogeneity and the MR‐Egger intercept test for pleiotropy, further validate our results by indicating no significant biases.^12^ To further validate the reliability of our findings, we referenced recent bidirectional Mendelian randomization analyses,^13^ which found no causal relationship between psoriasis and bladder cancer, and similarly confirmed no causal association between atopic dermatitis and COVID‐19 outcomes.^14^

However, our study is not without limitations. The GWAS datasets used were derived from European populations, which may limit the generalizability of our findings to other ethnic groups. Although we rigorously selected genetic variants as instrumental variables based on genome‐wide significance and linkage disequilibrium, there is always a potential for weak instruments to introduce bias. Nonetheless, our sensitivity analyses suggest that this is unlikely to have significantly affected our results.

The absence of a causal relationship between HPV and SLE in our study might suggest that other environmental or genetic factors play a more significant role in the pathogenesis of SLE.^15^, ^16^, ^17^, ^18^, ^19^ Alternatively, it is possible that the impact of HPV on autoimmune responses is complex and involves mechanisms not captured by our genetic instruments. Further research exploring these mechanisms at a molecular level could provide additional insights.

Future studies should consider exploring other viral infections and their potential links to autoimmune diseases using similar robust methodological approaches. Expanding the study to include diverse populations could help to understand the role of genetic and environmental interactions in the development of SLE. Additionally, integrating multi‐omics data, such as transcriptomics and proteomics, could provide a more comprehensive understanding of the biological pathways involved.^20^, ^21^, ^22^

In conclusion, our bidirectional two‐sample MR analysis indicates no causal relationship between HPV infection and SLE. These findings contribute to the growing body of literature on the etiology of SLE and highlight the importance of using robust epidemiological methods to clarify complex disease relationships. Further research is necessary to explore other potential risk factors and to elucidate the underlying mechanisms of autoimmune diseases.

## 5 CONCLUSIONS

Our two‐way two‐sample MR Analysis showed no causal relationship between HPV infection and SLE. These findings contribute to the growing literature on the etiology of systemic lupus erythematosus and underscore the importance of using robust epidemiological approaches to elucidate complex disease relationships.

## CONFLICT OF INTEREST STATEMENT

All authors declare that there are no conflicts of interest regarding the content of this article. Additional information can be found in the supplementary files.

## ETHICS STATEMENT

The ethics of this article are in the original data article.

## Supporting information

Supplement Table S1 SNPS in HPV16/18

## Data Availability

The datasets presented in this study can be found in online repositories.
